# Prediction of Scar Myometrium Thickness and Previous Cesarean Scar Defect Using the Three-Dimensional Vaginal Ultrasound

**DOI:** 10.1155/2022/3584572

**Published:** 2022-10-05

**Authors:** Liang Shi, Keke Du

**Affiliations:** ^1^Department of Gynaecology and Obstetrics, Xinchang People's Hospital, Shaoxing 312500, Zhejiang Province, China; ^2^Department of Gynaecology and Obstetrics, Wenzhou Central Hospital, Wenzhou 325000, Zhejiang, China

## Abstract

This research aimed to explore the related factors of scar myometrial thickness and scar diverticulum formation and then predict the occurrence of uterine diverticula. 140 patients with cesarean section were selected as the research objects. According to the three-dimensional (3D) vaginal ultrasound echo and the diagnostic criteria of uterine diverticulum, the research objects were divided into a diverticulum group and a control group, with 70 cases in each group. Data such as age, number of cesarean sections, endometrial thickness, uterine position, and diverticulum size was collected, and their relationship with uterine diverticulum was compared and analyzed. The results showed that there were significant differences in menstrual days, cesarean section times, and uterine position between the two groups (*P* < 0.05). The height (9.02 ± 2.97), width (14.02 ± 3.08), and depth (5.14 ± 1.23) of the posterior uterine diverticula in the scar diverticulum group were all greater than the anterior uterine height (6.69 ± 1.36), the width (10.69 ± 2.15), and the depth (3.86 ± 0.69), respectively. The residual myometrium thickness in posterior position of the uterus (2.98 ± 0.75) was < anterior position of uterus (3.43 ± 0.47), and the difference was statistically significant (*P* < 0.05). Multivariate analysis showed that the frequency of cesarean section (1 time, 2 times), uterine position, and abnormal menstruation were independent risk factors in the scar diverticulum group (*P* < 0.05). In conclusion, menstrual abnormalities, the number of cesarean sections (1 time or twice), and the position of the uterus are independent risk factors for the formation of uterine scar diverticula. The deeper the diverticula, the more likely to have menstrual abnormalities, the more prone to diverticulum in patients with posterior uterus, and the deeper the diverticula in patients with 2 dissections.

## 1. Introduction

A cesarean section is an abdominal incision of the uterus to remove a viable fetus [1]. It is different from the birth canal in that the fetus does not pass through the mother's vagina, but directly cuts the uterus through the abdomen through surgery and then removes the fetus from the uterus, which is an important operation in the field of obstetrics and gynecology [2]. With the continuous progress of scientific and technological level and medical level, the subject knowledge related to surgery has become more systematic and perfect, the surgical equipment has become more advanced, and the surgical methods and required materials have also been greatly improved. Based on the above advantages and progress, cesarean section technology has been applied and promoted in clinical practice and has become an important means for obstetricians to treat mothers and fetuses. Under normal circumstances, pregnant women can give birth through the vagina, but some pregnant women cannot guarantee the smooth delivery of the fetus due to their small pelvis. Due to pathological reasons, the fetus is too large, abnormal fetal development, placental abruption, etc., endanger the safety of the fetus and the mother. If the pregnancy needs to be terminated early, the delivery will be terminated by cesarean section [3, 4]. Cesarean section operation is traumatic to a certain extent, so the puerperae should do a good job of cleaning the wound after the operation and disinfecting the clothes and the ward environment to avoid wound infection [5]. Cesarean section, as an obstetric method for dealing with dystocia and high-risk pregnancies, can reduce maternal and perinatal mortality and reduce serious childbirth complications [6]. In the past 20 years, the rate of cesarean section at home and abroad has been increasing. The average rate of cesarean section in our country in 2011 was 54.47%, and the highest area was 71.59%; cesarean section without indication accounted for 26.51% [7]. As the rate of cesarean section increases, the long-term complications after cesarean section also increase year by year, among which the incidence of uterine scar diverticulum after cesarean section is 19.4 to 88.0% [8].

After cesarean section, the wound will heal and produce uterine scar, but poor healing will produce previous cesarean scar defect (PCSD) [9]. Poor wound healing leads to thinning of the muscle layer at the uterine scar, forming a depression or lacuna that communicates with the uterine cavity [10, 11]. The causes of PCSD can be divided into two sources: one is caused by congenital defect or abnormal embryo development; the second is caused by acquired external factors, among which the poor healing effect of the myometrium after cesarean section is the main reason [12]. According to statistics, the rate of cesarean section in China is as high as 46.2%, and the corresponding incidence of uterine PCSD also increases. Most patients with uterine PCSD will have abnormal uterine bleeding, and the probability of abnormal uterine bleeding after cesarean section is as high as 89% [13, 14]. Abnormal uterine bleeding may lead to decreased chances of successful pregnancy and even infertility, dysmenorrhea, chronic pelvic pain, and other symptoms, which to a certain extent have a great negative impact on the patient's physical and psychological. Once diverticulum pregnancy or scar pregnancy occurs, it can lead to dangerous placenta implantation, uterine split, and massive bleeding, even endanger the lives of mothers and children, and lead to adverse maternal and infant outcomes [15, 16].

At present, the examination of uterine diverticulum mainly includes ordinary transabdominal and transvaginal two-dimensional color Doppler ultrasound, three-dimensional transvaginal ultrasound (TVUS), hysterography (SHG), magnetic resonance imaging (MRI), and hysteroscopy [17]. Uterine contrast-enhanced ultrasonography can well observe the existence of scarred diverticulum, but it cannot measure the size of the diverticulum, and some people are allergic to contrast agents. Hysteroscopy can clearly display the presence or absence of scar diverticulum under the microscope, observe the shape and blood flow of the diverticulum, and can also repair the scar diverticulum at the same time, but as an invasive operation, hysteroscopy is not suitable as a screening method. Compared with two-position ultrasound, three-dimensional ultrasound can observe the three-dimensional spatial structure of scar and observe the shape, volume, and blood flow parameters of scar diverticulum [18, 19]. Therefore, in this work, three-dimensional vaginal ultrasound was selected to detect patients who had more than one cesarean section experience and to observe and record the residual thickness of the myometrium. In addition, it analyzes the relationship between factors such as patient age, uterine position, number of cesarean sections, and the formation of uterine scar diverticulum, to summarize the rules, hoping to provide a certain reference value for clinical prediction of the occurrence of scar diverticulum.

## 2. Materials and Methods

### 2.1. Research Objects

One hundred and forty patients who visited hospital from January 2018 to January 2021 and had one or more cesarean sections were selected as the research objects. According to the echo of 3D TUVS and the diagnostic criteria of uterine PCSD and uterine scar integrity [20], subjects were divided into a PCSD group and the uterine scar integrity group (namely the control group), with 70 cases in each group. This study had been approved by the ethics committee of hospital. All the patients and their families had agreed to sign corresponding informed consent forms.

Inclusion criteria are as follows: patients with at least one history of cesarean section and the surgical method was lower uterine cesarean section; age range: 20 to 45 years; and the first visit and had not received systematic treatment.

Exclusion criteria are as follows: patients with abnormal uterine bleeding due to endometrial polyps, submucosal fibroids, endocrine abnormalities, and other reasons; patients who were pregnant again; patients suffering from systemic diseases; and patients with vaginal examination, incomplete data, or unable to complete the whole process of the experiment.

### 2.2. Experimental Methods

The experimental subjects were examined by transvaginal color Doppler ultrasound to observe the echoes of the experimental subjects' uterine scars, and the subjects were divided into scar diverticulum group and scar integrity group according to whether there were irregular anechoic areas. In the scar diverticulum group, after the image was properly enlarged during the measurement of the diverticulum, the long diameter (upper and lower diameter) and depth of the scar diverticulum were measured on the longitudinal section of the uterus, and then, the transverse diameter (wide diameter) of the diverticulum was measured on the transverse section rotated by 90°. Finally, the image was fully enlarged, and the thickness of the residual myometrium in the anterior wall of the uterus at the diverticulum was measured at the maximum depth of the anechoic dark area on the longitudinal section of the uterus. The specific measurement of each diameter line is based on the upper and lower diameter of the scar defect: the distance from the base of the echo-free area along the longitudinal axis of the uterus on the longitudinal section; scar defect depth: the vertical distance from the top to the base of the anechoic zone on the longitudinal section; residual myometrial thickness: the distance from the top of the anechoic zone on the longitudinal section to the uterine serosa at this level; the thickness of the adjacent myometrium: the thickness of the complete myometrium near the fundus of the uterus in the anechoic area on the longitudinal section; and left and right diameter of scar defect: the width of the echo-free area on the transverse section. The patient's basic information, endometrial thickness, uterine position, and measurement data of diverticula were collected, and related factors were analyzed. The specific process is shown in Figure 1.

### 2.3. Examination by 3D TUVS

The complete sonographic image of scar showed the transverse indentation of the myometrial echo at the lower segment of the anterior uterine wall of the cesarean section scar, or saw a linear hyperechoic or hypoechoic area connecting the two sides of the muscle layer, and no obvious anechoic area was found under the muscle layer. The sonogram of scar diverticulum showed continuous serosal echo at the lower segment of the cesarean section scar of the anterior uterine wall, partial echo interruption of the muscle layer, incomplete endometrial continuity, and wedge-shaped, triangular, or irregular anechoic areas under the muscle layer. The width, height, and depth of the diverticulum were measured from the longitudinal and transverse sections of the uterus, respectively, and then, the thickness of the residual myometrium in the anterior uterine wall of the diverticulum was measured at the maximum depth of the anechoic dark area on the longitudinal section of the uterus. The specific measurement methods are shown in Table 1.

### 2.4. Observation Indexes

General information of patients included age, endometrial thickness, menstrual days, number of cesarean sections (1, 2, 3), and uterine position (anterior, posterior); measurement data of scar diverticulum include width, height, depth, and thickness at the thinnest part of the remaining myometrium.

### 2.5. Statistical Methods

SPSS 22.0 statistical software package was used for statistical analysis. Measurement data were expressed as mean ± standard deviation, the independent-samples *t*-test was used for intergroup data, the chi-square analysis and rank-sum test were used for nonparametric test of enumeration data, and unconditional logistic regression analysis was used for independent factors of PCSD. *P* < 0.05 considered the difference to be statistically significant.

## 3. Results

### 3.1. General Data

Analysis on basic data of patients revealed that there was no significant difference in age and endometrial thickness between two groups (*P* > 0.05). The differences in menstrual days and the number of cesarean sections were statistically significant (*P* < 0.05). The patients in PCSD group had significantly more menstrual days than those in the control group, and the difference was statistically significant (*P* < 0.05). The details are shown in Table 2. The number of cesarean sections in the PCSD group was larger than that in the control group, and Table 3 shows that the ratio of patients with two cesarean sections in the PCSD group was 45.71%, which was larger than the ratio of 18.57% in the control group. The difference in uterine position between two groups was statistically significant (*P* < 0.05). The patients with posterior uterus accounted for 70% in the PCSD group and those with anterior uterus accounted for 65.71% in the control group, and the difference was statistically significant (*P* < 0.05).

### 3.2. Relationship between Menstrual Abnormalities and Various Measurement Data of Scar Diverticulum in the Scar Diverticulum Group

There were no significant differences in the height, width, and remaining myometrium thickness in the thinnest location between normal and abnormal menses in the PCSD group (*P* > 0.05). The difference in the depth of PCSD was statistically significant (*P* < 0.05). The depth of PCSD of patients with abnormal menstruation (6.34 ± 2.02) was significantly greater than that of patients with normal menstruation (4.65 ± 1.68). The details are shown in Figure 2 and Table 4.

### 3.3. The Relationship between the Position of the Uterus and the Measurement Data of the Scar Diverticulum in the Scar Diverticulum Group

There were statistically significant differences in the height, width, and depth of the scar diverticulum between the anterior and posterior uterine position of the PCSD group (*P* < 0.05). The thickness of the thinnest residual myometrium in patients with anterior uterus was 3.43 ± 0.47 mm significantly larger than that in patients with posterior uterus (2.98 ± 0.75 mm), as shown in Figure 3 and Table 5.

### 3.4. Relationship between the Frequency of Cesarean Section and the Measurement Data of Scar Diverticulum in the Scar Diverticulum Group

There was no significant difference in the number of cesarean sections and the height and width of the diverticulum in the scar diverticulum group (*P* > 0.05). There were statistically significant differences in the number of cesarean sections, the depth of diverticulum, and the thickness of residual myometrium (*P* < 0.05). Among them, with the increase in the number of cesarean sections, the depth of the diverticulum increased, and the thickness of the residual myometrium decreased, and the difference was statistically significant (*P* < 0.05). The details are shown in Figure 4 and Table 6.

### 3.5. Multivariate Analysis of Factors Related to the Formation of Scar Diverticulum

Multivariate analysis was performed for categories with *P* < 0.05 in univariate analysis. The results showed that menstrual abnormalities, uterine position (anterior position, posterior position), and 1 and 2 cesarean sections were independent factors for the occurrence of scar diverticulum (*P* < 0.05). The details are shown in Table 7.

## 4. Discussion

Cesarean section is an important surgical method for obstetric treatment of pregnant women and their fetuses by cutting open the abdomen and uterus of pregnant women and removing the fetus from the uterus. The application of cesarean section is mainly aimed at the pregnant women with fetal intrauterine distress, delayed labor, pelvic stenosis, abnormal fetal position, multiple pregnancy or previous pregnancy with a history of cesarean section, placenta previa, or too large fetus to deliver through the vagina. This greatly reduces the risk index of childbirth for mothers and fetuses who are not suitable for natural delivery [21]. Scar diverticulum is a complication following cesarean section and is a defect formed by poor uterine incision healing [22]. Patients with uterine scar diverticulum are mainly manifested as prolonged, incessant menstruation and lower abdominal pain after cesarean section, causing secondary infertility [23]. Most patients with small diverticula do not have any clinical symptoms. However, some women will experience abnormal bleeding during non-menstrual period for a long time, prolong the menstrual cycle, and even cause anemia [24]. This has a certain impact on the patient's health and quality of life. Therefore, understanding the relevant disease characteristics of patients with uterine scar diverticulum and sorting out and analyzing to find the rules may provide a reference for clinical prediction of the occurrence of uterine scar diverticulum in advance [25].

A large number of studies have shown that the formation of uterine scar diverticula after cesarean section is closely related to the posterior position of the uterus [26, 27]. Early studies by foreign scholars found that the probability of uterine scar diverticulum after cesarean section in the posterior uterus is twice that of the anterior uterus. In this work, the multivariate analysis showed that menstrual days and uterine position were independent risk factors for the occurrence of diverticula, and the results were similar. It was found that the width, height, and length of the scar diverticulum in the abnormal menstrual group were greater than those in the normal menstrual group. It is suggested that the width, height, and length of scar are related to abnormal uterine bleeding. In this study, the measurement values of each diameter of patients with abnormal menstruation in the PSCD group were height (6.07 ± 2.45 mm), width (9.13 ± 4.63 mm), and depth (6.34 ± 2.02 mm); the measured diameters of normal menstrual patients were 6.40 ± 2.32 mm in height, 9.18 ± 3.84 mm in width, and 4.65 ± 1.68 mm in depth. At the same time, there was no significant difference in height, width, and thickness of the thinnest part of the remaining muscle layer in the measured values of PCSD between patients with abnormal menstruation and normal menstruation (*P* > 0.05). Only the depth difference was statistically significant (*P* < 0.05). It is suggested that the deeper the diverticula, the more likely to have abnormal menstruation, and the results are similar. Due to the increased depth of the diverticulum, there is a greater likelihood of accumulation of blood in the diverticulum, thereby predisposing to abnormal vaginal bleeding and possibly longer duration of bleeding. A comparison of the uterine position of the two groups of patients suggested that the PSCD group had the most posterior uterus, accounting for 70%, and the control group had 65.71% anterior uterus; the difference was statistically significant (*P* < 0.05). This indicates that women with a posterior uterus are more likely to develop uterine scar diverticula after cesarean section. In existing studies, it has also been shown that the generation of uterine scar diverticula after cesarean section is closely related to the posterior position of the uterus [28]. Early scholars found that women with cesarean section experience are more likely to develop uterine scar diverticula after surgery [29], and the probability of occurrence is twice that of women with anterior uterus [30]. It is consistent with the results of this work. At the same time, in the comparison of the uterine position and the measured values of the diverticulum, it was found that the height of the posterior uterine diverticula was 9.02 ± 2.97 mm, the width was 14.02 ± 3.08 mm, and the depth was 5.14 ± 1.23 mm, which were all greater than the height of the anterior uterus by 6.69 ± 1.36 mm, width by 10.69 ± 2.15 mm, and depth by 3.86 ± 0.69 mm. The thickness of the thinnest residual myometrium was 2.98 ± 0.75 in the posterior uterus and 3.43 ± 0.47 in the anterior uterus. The posterior uterus was thinner than the anterior uterus, and the above was statistically significant (*P* < 0.05). This indicates that the diverticulum in the posterior uterus is more serious than that in the anterior uterus. It is considered that when the uterus is retroverted and flexed, the tension of the muscle layer significantly expands and pulls the wound, resulting in poor wound cohesion, incomplete healing surface, and the appearance of diverticula. The diverticulum thickness of the patients with 2 cesarean sections in the PSCD group was greater than that of the patients with 1 cesarean section, and multivariate analysis was performed for the category of *P* < 0.05 in the univariate analysis. The results showed that 1 and 2 cesarean sections were independent factors for the occurrence of scar diverticula, indicating that the more cesarean sections, the thicker the diverticula. Three times of cesarean section is not a relevant risk factor. The fertility policy and clinical practice of China will take the measure of strengthening suture in patients with more than two cesarean sections, so as to reduce the production of diverticulum.

## 5. Conclusion

The results of this work indicated that menstrual abnormalities, the number of cesarean sections (1 time, 2 times), and uterine position were independent risk factors for the formation of uterine scar diverticula. The deeper the diverticula, the more likely to have abnormal menstruation. Compared with the anterior uterus, the posterior uterine diverticulum was more serious, and the diverticulum thickness of the patients with two cesarean sections was greater than that of the patients with one cesarean section. However, the research time and sample size of this study were limited. In the future, if conditions are permitted, large-scale, multicenter, and multiregional studies may be more convincing.

## Figures and Tables

**Figure 1:** Technology routine.

**Figure 2:** PCSD size with normal and abnormal menstruation. (a) The patient with normal menstruation and (b) the diameter value of the patient with abnormal menstruation. H, W, D, and R referred to height, width, depth, and remaining myometrium thickness, respectively.

**Figure 3:** PCSD size with posterior and anterior uterine position. (a) Uterus anterior and (b) uterus posterior. H, W, D, and R referred to height, width, depth, and remaining myometrium thickness, respectively.

**Figure 4:** Relationship between the number of cesarean sections and PCSD size. (a) 1 cesarean section; (b) 2 cesarean sections; (c) 3 cesarean sections; (d) change trend of the measured values of each diameter with the increase in cesarean sections. H, W, D, and R referred to height, width, depth, and remaining myometrium thickness, respectively.

**Table 1:** Measurement methods of each data of PCSD.

Parameter	Measurement methods
Width	Maximum distance between left and right diameter lines of anechoic zone on 3D longitudinal section of uterus

Height	Maximum vertical distance between upper and lower diameter lines of anechoic zone on longitudinal section of uterus 3D image

Depth	The maximum distance from the tip of anechoic zone to the base on the transverse section of transvaginal two-dimensional image

The remaining myometrium thickness in the thinnest location	Minimum distance from the top of anechoic zone on longitudinal section to the serosal layer on horizontal plane

**Table 2:** Comparison on basic data of patients in two groups.

Item	Group		t	*p*
	PCSD group	Control group		
Age (years old)	34.12 ± 2.58	39.88 ± 4.59	2.044	0.532
Endometrial thickness (mm)	5.37 ± 1.12	5.50 ± 1.94	0.565	0.603
Menstrual days (days)	5.58 ± 1.51	11.84 ± 3.15	3.618	0.000
The number of cesarean sections (times)	1.22 ± 0.47	1.57 ± 0.46	3.618	0.000

**Table 3:** Comparison on the number of cesarean sections and uterine position.

Item		PCSD group (70 cases)		Control group (70 cases)		*x* ^2^	*p*
		Cases	Proportion (*n*%)	Cases	Proportion (*n*%)		
The number of cesarean sections (times)	1	34	48.57	55	78.57	13.121	0.003
	2	32	45.71	13	18.57		
	3	4	5.71	2	2.86		

Uterine position	Anterior	21	30.00	46	65.71	16.375	0.000
	Posterior	49	70.00	24	34.29		

**Table 4:** Relationship between PCSD diameter measurements and menstrual abnormalities (mm).

Menstrual condition	Measurement data of each diameter line of PCSD			
	Height (mm) (up and down diameter)	Width (mm) (left and right diameter)	Depth (mm)	The thickness of the thinnest part of the remaining muscle layer (mm)
Abnormal menstruation	6.07 ± 2.45	9.13 ± 4.63	6.34 ± 2.02	3.44 ± 1.76
Normal menstruation	6.40 ± 2.32	9.18 ± 3.84	4.65 ± 1.68	3.53 ± 1.09
*T* value	0.316	0.033	−3.154	0.212
*p*	0.697	0.984	0.002	0.932

**Table 5:** Relationship between PCSD diameter measurements and menstrual abnormalities (mm).

Menstrual condition	Measurement data of each diameter line of PCSD			
	Height (mm) (up and down diameter)	Width (mm) (left and right diameter)	Depth (mm)	The thickness of the thinnest part of the remaining muscle layer (mm)
Abnormal menstruation	6.07 ± 2.45	9.13 ± 4.63	6.34 ± 2.02	3.44 ± 1.76
Normal menstruation	6.40 ± 2.32	9.18 ± 3.84	4.65 ± 1.68	3.53 ± 1.09
*T* value	0.316	0.033	−3.154	0.212
*p*	0.697	0.984	0.002	0.932

**Table 6:** Relationship between PCSD diameter measurements and the number of cesarean sections (mm).

The number of cesarean sections (times)	Measurement data of each diameter line of PCSD			
	Height (mm) (up and down diameter)	Width (mm) (left and right diameter)	Depth (mm)	The thickness of the thinnest part of the remaining muscle layer (mm)
1	6.65 ± 2.59	10.34 ± 4.13	4.37 ± 1.87	4.25 ± 1.36
2	6.32 ± 2.68	9.07 ± 3.97	5.68 ± 1.75	3.34 ± 1.25
3	4.87 ± 3.25	6.56 ± 4.21	7.91 ± 1.69	2.79 ± 0.41
*T* value	1.601	1.361	9.483	11.324
*p*	0.452	0.916	0.000	0.000

**Table 7:** Results of multivariate analysis for the occurrence of scar diverticula.

Relevant factors	Regression coefficients	Standard error	Wals value	*P*	OR	95% CI
Normal menstruation	1.561	0.514	0.702	0.521	0.712	0286–16.265
Abnormal menstruation	2.037	0.293	8.428	0.002	4.179	4.245–12.749
1 cesarean section	1.648	0.496	2.032	0.169	2.121	0.818–5.615
2 cesarean sections	1.765	0.567	8.960	0.004	5.310	1.763–16.117
3 cesarean sections	1.534	0.779	3.726	0.063	4.362	0.998–19.332
Anterior uterus	1.964	0.391	6.141	0.015	2.62	1.321–5.679
Posterior uterus	1.816	0.395	20.014	0.001	5.814	2.813–13.359

## Data Availability

The data used to support the findings of this study are available from the corresponding author upon request.
